# English Grammar Detection Based on LSTM-CRF Machine Learning Model

**DOI:** 10.1155/2021/8545686

**Published:** 2021-08-17

**Authors:** Liqin Wu, Meisen Pan

**Affiliations:** ^1^School of International Education, Hunan University of Medicine, Huaihua, Hunan 418000, China; ^2^College of Computer and Electrical Engineering, Hunan University of Arts and Science, Changde, Hunan 415000, China

## Abstract

Deep learning and neural network have been widely used in the field of speech, vocabulary, text, pictures, and other information processing fields, which has achieved excellent research results. Neural network algorithm and prediction model were used in this paper for the study and exploration of English grammar. Aiming at the application requirements of English grammar accuracy and standardization, we proposed a machine learning model based on LSTM-CRF to detect and analyze English grammar. This paper briefly summarized the development trend of deep learning and neural network algorithm and designed the structure pattern of radial basis function neural network in grammar semantic detection and analysis on the basis of deep learning artificial neural network theory. Based on the morphological features of English grammar, a grammar database was established according to the rules of English word segmentation. In this paper, we proposed an improved conditional random field CRF (Conditional Random Field) network model based on LSTM (Long Short-Term Memory) neural network. It can improve the problem that the traditional machine learning model relies on feature point selection in English grammar detection. The machine learning model based on LSTM-CRF was used to recognize English grammar text entities. The results show that the English grammar detection system based on the LSTM-CRF model can simplify the process structure in the recognition process, reduce the unnecessary operation cycle, and improve the overall detection accuracy.

## 1. Introduction

The research of artificial neural networks is one of the important contents in the field of intelligent science and technology. It is also the basic rudiment of deep learning neural network structure. In the exploration of neural network structure analysis and mechanism, researchers have constructed similar network structures [1]. It can make the computer model get a large number of learning data in the process of training for law analysis. In the last century, researchers took the lead in developing the perception ability in the model mechanism and put forward the mathematical model of artificial neural network structure [2]. Subsequently, the invention of the inversion algorithm puts the research of artificial neural network into a fanatical stage. Due to the lack of a comprehensive understanding of the algorithm and network structure, theoretical analysis is difficult. The learning and training methods and technologies are not perfect. When the structure of the artificial neural network has just become the focus of the world, the development of computer science is not strong enough [3]. Because the computing speed and accuracy of the computer cannot meet the requirements of the neural network structure at that time, therefore, the structure of the neural network in this period is relatively simple, and most of its internal structure is composed of single-level neurons, mainly providing shallow learning and training research [4].

With the development of science and technology and the progress of the computer field, the structure of the neural network is constantly updated. Subsequent researchers proposed the method of layer-by-layer expected training, which significantly improved the accuracy of language recognition [5]. At this stage, the thought and research direction of deep learning was officially opened [6]. In the research of deep learning structure, from the experimental data of image processing, language recognition, text detection, pattern detection, and so on, it is more suitable for learning training models than the traditional neural network algorithm [7]. This also proves that deep learning has great advantages and status in neural network structure [8], from the single neural network unit structure to the multilevel neural network structure under deep learning. The complexity of network structure makes the number of layers and variables increasing, which increases the range of data sources. It can find more data feature points in the range of data sources and obtain excellent learning and training effect [9].

With the continuous development of deep learning theory, it has been pursued by more and more researchers. With the growth of computing power and detection technology, this model has been used in many fields [10]. Microsoft researchers improved the accuracy of speech recognition by using deep learning neural network algorithm, which reduced the recognition error rate by two to three percentage points [11]. Then, in the aspect of pattern recognition and data detection, the difference of detection results is reduced by 15%. Compared with the traditional algorithm, deep learning neural network algorithm can reduce the prediction model and recognition error [12].

The English language is one of the common languages in various fields of scientific research and cooperation. For the use of English grammar, each country has its own characteristics [13]. For example, there are obvious differences in English grammar. There are also grammatical and semantic differences among states and cities in the same country [14]. How to detect and analyze English grammar intelligently is a basic technology in simultaneous translation and English writing [15]. By improving the ambiguity between English grammar and semantics, we can improve the efficiency of English reading, communication, and communication. In the actual detection operation, the semantic character and recognition effect will be affected [16]. It seriously interferes with the optimization test and detection efficiency of English grammar. Based on the above problems, we propose to use the LSTM-CRF machine learning model to calculate English grammar detection data and build the model [17]. LSTM neural network is long short memory neural network, and CRF neural network is conditional random field algorithm. According to the combination of the features of the two algorithms, the classification can be accurately distinguished according to the semantic and grammatical relationship between the upper and lower texts [18]. Finally, the purpose of data analysis and detection is achieved. The LSTM-CRF neural network algorithm is used to label the English text and define the sample [19]. In the process of finding different feature points, we compare the advantages and disadvantages of the model with the traditional algorithm [20]. In the process of English grammar detection, we need to explore the way of text recognition. We use the optimized algorithm after the combination of the two to study the entity recognition of English text [21]. At the same time, according to the training model formed by the combination of LSTM neural network algorithm and CRF neural network algorithm, English grammar detection and analysis are carried out, and the advantages of this algorithm in data simulation and data analysis are obtained [22]. With the combination of the two, the network has been applied to realize the establishment of English speech recognition and translation, word feedback and machine learning, intelligent English grammar translation, and other models. This technical level is constantly updated and improved.

Firstly, this paper introduces the advantages and development of deep learning neural network algorithms and explores the intelligent analysis technology of semantics in English grammar based on neural network technology. Secondly, it studies the English grammar word segmentation technology under the LSTM-CRF machine learning model, mainly analyzing the CRF machine learning model. Finally, this paper studies the English grammar entity recognition technology based on LSTM-CRF machine learning, discusses the function of LSTM and CRF neural network layer, and finally analyzes the influence of the construction model of the combination of LSTM and CRF on grammar detection.

## 2. Research on English Grammar Detection Technology Based on Neural Network Algorithm and LSTM-CRF Model

### 2.1. English Grammar and Semantic Analysis Technology Based on Neural Network Algorithm

Aiming at the requirement of intelligent analysis of semantic content in English grammar detection, we study the automatic recognition function of English characters [23]. By using the basis function of neural network in the machine learning model, a method of English grammar character recognition based on a neural network algorithm is proposed [24]. The basic function of the neural network can replace the activation function of the traditional algorithm and improve the simulation effect of the whole network structure [25]. Learning training based on the gradient descent method can speed up the detection efficiency and performance of the model [26].

A neural network is the basic model building algorithm in the field of machine learning [27]. In order to improve the poor training effect caused by the complexity of the input data source in the traditional algorithm, we introduce the radial basis function neural network algorithm. This algorithm is used to replace the nonlinear variable in the traditional algorithm. Firstly, the structure of neurons in the neural network is briefly introduced [28]. An artificial neural network can imitate human brain activity according to the model memory and process information. It mainly involves the unit structure, network structure, network training, and other aspects. The basic structure of the neural network is shown in Figure 1.

The variables are defined in the figure represent input data and are connected by weight variables between unit nerves. Different input data and weight values are one-to-one correspondence. According to these variables, the weight matrix of the whole structure is generated. The output matrix is as follows:

(1) $$\begin{array}{c} y=f\left(x_{1}w_{r1}+x_{1}w_{r1}+\ldots +x_{n}w_{rn}-\theta_{r}\right),\\ y=f\left(\sum_{i=0}^{n}w_{ir}x_{r}-\theta_{r}\right). \end{array}$$

There is an activation function in the formula, and the process of function transformation is nonlinear. Using this method in the whole neural network can increase the simulation ability of network detection. Every single neuron forms a whole neural network structure according to the way of head tail combination. BP algorithm is basically used in model learning training, but this algorithm has no advantage in grammar and semantic analysis. In order to improve the above problems of the BP neural network, we introduce the radial basis function neural network algorithm. The basic structure of this neural network algorithm is consistent with that of a general neural network. They are input layer, output layer, and fading layer. Compared with the basic element structure, the radial basis function replaces the activation function of the basic element structure in the gradually hidden layer. The formula is as follows:

(2) $$\begin{array}{c} h_{j}=\exp\left(\frac{{\left\|x-c_{j}\right\|}^{2}}{2b_{j}^{2}}\right),\\ c=\left[c_{ij}\right]=\left[\begin{array}{ccccc} c_{11} & . & . & . & c_{1m}\\ . & . & \; & \; & .\\ . & \; & . & \; & .\\ . & \; & \; & . & .\\ c_{n1} & . & . & . & c_{nm} \end{array}\right],\\ b={\left[\begin{array}{ccc} b_{1}, & \ldots , & b_{m} \end{array}\right]}^{T},\\ y_{m}=\sum_{j}^{m}w_{j}h_{j}. \end{array}$$

In the above formula, *c* is the position of the function of the element of the *j* gradually hidden layer, *b* is the height of the calculated function. In order to make the actual output more close to the expected effect, we need to improve the parameters of the whole structure by learning and training the neural network model. In the radial basis function neural network algorithm, we determine the error variables in the overall network structure according to the gradient operation method. In this study, the mean variance is used to represent the error analysis variables. The calculation formula is as follows:

(3) $$\begin{array}{c} E\left(t\right)=\frac{1}{2}{\left(y\left(t\right)-y_{m}\left(t\right)\right)}^{2}. \end{array}$$

The weight value is updated, and the formula is as follows:

(4) $$\begin{array}{c} \Delta w_{j}\left(t\right)=-\gamma \frac{\partial E}{\partial w_{j}}=\gamma \left(y\left(t\right)-y_{m}\left(t\right)\right)h_{j}, \end{array}$$

(5) $$\begin{array}{c} w_{j}\left(t\right)=w_{j}\left(t-1\right)+\Delta w_{j}\left(t\right)+\delta \left(w_{j}\left(t-1\right)-w_{j}\left(t-2\right)\right). \end{array}$$

To update the width variable of the overall network structure, the calculation formula is as follows:

(6) $$\begin{array}{c} \Delta b_{j}\left(t\right)=-\gamma \frac{\partial E}{\partial b_{j}}=\gamma \left(y\left(t\right)-y_{m}\left(t\right)\right)w_{j}h_{j}\frac{{\left\|x-c_{j}\right\|}^{2}}{b_{j}^{3}}, \end{array}$$

(7) $$\begin{array}{c} b_{j}\left(t\right)=b_{j}\left(t-1\right)+\Delta b_{j}\left(t\right)+\delta \left(b_{j}\left(t-1\right)-b_{j}\left(t-2\right)\right). \end{array}$$

Finally, the central structure of the neural network is updated.

(8) $$\begin{array}{c} \Delta c_{ji}=-\gamma \frac{\partial E}{\partial c_{ji}}=\gamma \left(y\left(t\right)-y_{m}\left(t\right)\right)w_{j}h_{j}\frac{x-c_{ji}}{b_{j}^{2}}, \end{array}$$

(9) $$\begin{array}{c} c_{ji}\left(t\right)=c_{ji}\left(t-1\right)+\Delta c_{ji}\left(t\right)+\delta \left(c_{ji}\left(t-1\right)-c_{ji}\left(t-2\right)\right). \end{array}$$

In formulas (4) to (9), we define the learning efficiency and variable factors in the neural network model. Control these variables in a certain range. It is used to change the influence of the gradient of the model training learning process on the optimal solution. The whole process of training detection is shown in Figure 2.

In the flow chart, the whole neural network is initialized and defined according to the requirements, and the appropriate structure level is set. The model variables are propagated by way of data sample input. Compare the output data with the expected value and determine the difference between the two variables as the error analysis data. Finally, the whole network structure variables are updated until the output of the training process is closer to the expected results. When we study the effect in English grammar and semantic analysis, we can use the neural network structure to recognize English letters because of the patchwork nature of English letters, which is easier to manipulate than other languages. In the process of research, the corresponding characters in the range of 0 to 9 were selected. According to the digital generation method, it is expressed as a picture grid. The letter representation is shown in Figure 3.

As can be seen from Figure 3, the representation path of letter capitalization changes. Valid data is represented by 1 and invalid data by 0. For any different characters, we have corresponding different representation styles and finally arrange them in order. The above is the recognition process of grammar character digitization, which can improve the situation that the collected data is often interfered with by the irregular use of grammar in the process of grammar detection.

### 2.2. English Grammar Word Segmentation Technology Based on LSTM-CRF Machine Learning Model

In the process of English grammar testing, the English language needs to be processed by information technology. That is to say, we need to analyze the features of the language. Word segmentation is one of the basic tasks of data acquisition, data classification, detection, and analysis. Only after the word segmentation of English grammar is completed can the whole machine learning model be constructed. Most of the English writing methods use spaces as the separator, but the data set obtained by space segmentation changes the overall structure of the language. Based on the above situation, this paper proposes a segmentation process based on individual words. The commonly used word segmentation methods include traditional machine learning, deep neural network learning, and so on due to the limitations of traditional word segmentation, such as the storage of vocabulary number set, incomplete grammar rules, grammar conflict, and so on. At this time, we can construct word segmentation according to the CRF model. However, a single CRF algorithm model is easily limited by the design of a feature point template in the detection process. In the face of the range and way of collecting data feature points, the final results of the window combination we set in different syntax situations are different. In the follow-up, we add the word segmentation method based on the LSTM model and combine the advantages of the two to build the grammar detection model. We use LSTM level and CRF level to set syntax tags, which effectively improves the problem of feature point selection and input. The specific technical scheme is shown in Figure 4.

In the process of model vector construction, we need to transform the syntax text into variables. Every grammatical word is represented by a real variable. This method can reflect the semantic and grammatical relationship and improve the similarity of detection content in syntax detection. The specific syntax variable construction process is shown in Figure 5.

As shown in Figure 5, English sample sentences are divided into multimodule structures for classification research and set as interrelated variables. By dividing statements into different variables for detection, the running speed of the whole model can be improved.

In the establishment of the detection model, the long-term and short-term memory unit LSTM can improve the gradient disappearance problem in the traditional algorithm according to the selection unit gate. CRF algorithm can effectively extract the flag information in the whole grammar. The model based on LSTM-CRF can use the change data of time series to obtain feature points. The specific LSTM-CRF model is shown in Figure 6.

Let us take the grammar data monomer sample as an example: suppose there are 50 characters in the grammar, each of which is a variable of 25 dimensions. The feature point variables are constructed by characters, the output layer data is calculated, and the result matrix is obtained. Each LSTM neural network structure corresponds to a matrix. Finally, the matrix is input into the linear layer structure and marked according to the elements. All data are pieced together in a single character. The patchwork value is input into the CRF algorithm model, and the optimal data value in the detection result is obtained as the optimal solution of the detection model. The calculation formula of labeling process probability is as follows:

(10) $$\begin{array}{c} s\left(X,y\right)=\sum_{i=0}^{n}A_{y_{i},y_{i+1}}+\sum_{i=1}^{n}p_{t,y_{i}}. \end{array}$$

The formula after the optimization of the calculation results by likelihood estimation is as follows:

(11) $$\begin{array}{c} \log\left(p\left(y|X\right)\right)=s\left(X,y\right)-\text{lo}\underset{y\in Y_{x}}{\underset{∼}{g}}\text{adds}\left(X,y\right). \end{array}$$

After obtaining the best data result, the calculation formula of the optimal sorting path is as follows:

(12) $$\begin{array}{c} y^{*}=\text{ar}\underset{\underset{y\in Y_{x}}{∼}}{g}\max s\left(X,\tilde{y}\right). \end{array}$$

In the whole machine learning model, CRF level can constrain the unknown conditions by adding labels, which can improve the time complexity of detection results so as to ensure the effectiveness of grammar detection. The constraints in the LSTM-CRF machine model are obtained in the training process of CRF level, which improves the overall efficiency of English grammar detection.

### 2.3. Text Entity Recognition Technology for English Grammar Detection Based on LSTM-CRF Model

Text recognition of English grammar is to capture various variable labels in dynamic grammar changes. These variables can constitute a complex detection model. Therefore, this paper studies the text entity recognition technology in English grammar based on the neural network algorithm of the LSTM-CRF learning model. Combined with language processing, long-term and short-term memory neural network algorithm, and conditional random field algorithm, dynamic grammar change detection is studied. In the traditional entity recognition technology, we usually focus on three contents: variable, relation, and acquisition. Traditional algorithms include a single CRF entity recognition method. Firstly, the grammar database is constructed, and the characters are matched and segmented, and then the actual results are compared. Although this traditional single way is more efficient, it will be unable to capture when encountering problems such as huge data sources.

To solve the above problems, we propose a syntax entity recognition technology based on the LSTM-CRF machine learning model. It can plan variables and build a framework to avoid artificial interference and irregular interference. Firstly, we build the LSTM-CRF model according to algorithm rules, which mainly includes the LSTM level and CRF level. Bio word marking method is used to define the recognized grammatical sentences. The specific LSTM-CRF model is shown in Figure 7.

In the LSTM layer, we can see that there are several neural units, each unit is connected in series, and nonlinear motion is used to obtain the results in the whole detection process. The formulas of weight matrix and transfer vector are as follows:

(13) $$\begin{array}{c} i_{t}=\sigma \left(W_{i}∙\left[h_{t-1},x_{t}\right]+b_{i}\right),\\ f_{t}=\sigma \left(W_{f}∙\left[h_{t-1},x_{t}\right]+b_{f}\right),\\ o_{t}=\sigma \left(W_{o}∙\left[h_{t-1},x_{t}\right]+b_{o}\right),\\ \tilde{C_{t}}=\tanh\left(W_{c}∙\left[h_{t-1},x_{t}\right]+b_{c}\right),\\ C_{t}=f_{t}⊗C_{t-1}+i_{t}⊗\tilde{C_{t}},\\ h_{t}=o_{t}⊗\;\tanh\;C_{t}. \end{array}$$

In the calculation process, the LSTM model intelligently considers the change of variables in the same direction, and we can improve it to a two-way model to process the data information before and after. The variables calculated by the LSTM model are added to the CRF level for marking. At the CRF level, the results of the upper model can be constrained, and an optimal solution range can be controlled according to the marking relationship. The state change probability of the marked variable is calculated by the following formula:

(14) $$\begin{array}{c} s\left(X,Y\right)=\sum_{i=1}^{n}\left(a_{y_{i,}y_{i+1}}+p_{i,y_{i}}\right). \end{array}$$

The whole model construction is realized by a tensor flow algorithm. The model construction process is shown in Figure 8.

The syntax detection model based on the LSTM-CRF model can consider the overall detection process cost, time planning, efficiency, and other performance. Compared with the traditional model, it can better deal with complex data.

## 3. Result Analysis of Research Techniques in English Grammar Detection Based on LSTM-CRF Machine Learning Model

### 3.1. The Result Analysis of Neural Network Algorithm in English Grammar Detection Model

In order to more clearly distinguish the performance of neural network algorithms in the model, we carry out a comparative simulation test according to a variety of neural network algorithms. In order to ensure the equality of the test results, we set unified parameters for each variable in the test training. The specific parameters are shown in Table 1.

As shown in Table 1, we set the parameters of the number of hidden layers, the number of hidden units, the number of input and output nodes, and the maximum training times. This method effectively stabilizes the range of test results.

In the detection training, the test data variables are controlled according to the function, and the error rate index changes in the test are reflected by analyzing the curve changes in the ideal state and the state disturbed by the irregular grammar. The curve of irregular grade change and training recognition error rate is shown in Figure 9.

We can see that, according to the increase of irregular grammar, the greater the error rate of detection and recognition. Therefore, in the case of the same index variables, the rules of grammar have a certain influence on the overall English grammar detection results.

### 3.2. Analysis of Word Segmentation in English Grammar Detection Based on LSTM-CRF Model

The data sources used in the study are based on English Dictionary texts. According to the ratio of nine to one, the whole classification is divided randomly into training model and test model. We compare the traditional CRF model and the LSTM-CRF model. In the data source, the binary model is used to construct the amount of adjacent character transfer for text cutting. Due to the existence of a variable and distance relationship in English grammar, the appearance of characters and the relationship between them have an impact. The binary method cannot improve this problem, so we use the combination of long-term memory network algorithm and conditional random field algorithm. It can learn and train the time series information in the detection model and extract the feature points to improve the accuracy of the detection model.

In order to ensure the detection simulation structure has the optimal solution, we optimize the weights and migration variables according to the optimization function. The optimized training data is consistent with the output of the model as much as possible. We use the LSTM-CRF model for character embedding, and the dimensions are 25 and 50, respectively. The experimental results of the whole model are shown in Figure 10.

According to the experimental results, the long-term and short-term memory network algorithm inputs English grammar data in order and then sorts them in order and analyzes their historical influence. The LSTM algorithm is used to provide the best feature points for the CRF algorithm. The unlabeled variables of the experimental data are trained and learned and input into CRF level as feature results for marking. Finally, in the combined algorithm model, the detection effect is better than that of traditional CRF.

### 3.3. Result Analysis of Text Entity Recognition Technology for English Grammar Detection Based on LSTM-CRF Model

In order to clarify the applicability of the LSTM-CRF algorithm model and its role in each level, we detect dynamic syntax text in LSTM, CRF, and LSTM-CRF structure models, respectively. According to the accuracy, return efficiency and *F*1 index, the experimental results were analyzed as shown in Table 2.

According to Table 2, the CRF layer is mainly used to optimize processing according to all the statistical marker variables and receiving LSTM level output data. In training, we can use a rule algorithm to select grammar variables and adjust the changes between the parameters. After adding the CRF layer, the accuracy and return efficiency of the LSTM model can be changed. The significant changes in the accuracy and return efficiency in the table also confirm the role of CRF level in the detection model. Compared with the single LSTM model, the network model with conditional random field structure can better mediate the syntax detection process. The accuracy and efficiency of the whole model detection are improved.

In this study, the LSTM-CRF model is used to change the process of detection mark transformation according to the training learning results. The actual detection results are related to whether the label has the connection reaction. Firstly, the LSTM layer is used to train the detection function, and then the output results are obtained by changing the marking matrix according to the CRF marking function. It can be learned that the detection and recognition effect of the LSTM-CRF learning model can improve the accuracy and feedback efficiency.

## 4. Conclusion

With the continuous development of intelligence, in the use of general language, whether grammar is standard or not has a great influence on communication. Therefore, we need a faster, intelligent, and accurate English grammar model to reduce the cost of communication. This paper studies the role of neural network algorithms in the construction of the English grammar detection model and concludes that neural network algorithms can improve the efficiency of detection network training and can improve the performance of grammar character recognition. This paper uses LSTM-CRF machine learning to build a grammar word segmentation model to introduce and study the function of vocabulary in English grammar detection. This paper introduces the long-term and short-term memory neural network and conditional random field model to study the grammar segmentation and proves the superiority of the LSTM-CRF model in grammar detection. Finally, the performance of the CRF algorithm, LSTM algorithm, and LSTM-CRF combined algorithm in text entity recognition is compared and analyzed. The results show that the combined model can improve the efficiency of grammar detection, change the process of parsing grammar, reduce unnecessary links, and improve the overall performance. The experimental results show that the LSTM-CRF model can improve the accuracy and feedback speed of English grammar detection. In the construction of the English grammar detection model, this paper proposes to use the LSTM-CRF model to improve the detection efficiency and detection scope.

## Figures and Tables

**Figure 1:** Neural network infrastructure diagram.

**Figure 2:** Flow chart of training and testing process.

**Figure 3:** Letter representation method diagram.

**Figure 4:** Specific technical scheme diagram.

**Figure 5:** Syntax variable construction diagram.

**Figure 6:** LSTM-CRF model diagram.

**Figure 7:** LSTM-CRF model.

**Figure 8:** Flow chart of model construction.

**Figure 9:** Curve graph of irregular grade change and training recognition error rate.

**Figure 10:** Experimental results of LSTM-CRF model.

**Table 1:** Specific parameter.

Parameter name	Parameter value
Number of hidden layers	1
Number of hidden units	500
Number of input nodes	35
Number of output nodes	52
Target error	0.0001
Maximum training times	40

**Table 2:** Experimental comparison results.

Model	Accuracy	Return efficiency	*F*1 index
LSTM	0.796	0.787	0.791
CRF	0.859	0.805	0.831
LSTM-CRF	0.862	0.856	0.859

## Data Availability

All the data of this study are from the big data statistics of the test process. The data of this paper can fully support the research results of this paper.
